The article "CELL PROLIFERATION AND CYTOKINE INDUCTION BY TNF-α OF PSORIATIC KERATINOCYTES ARE NOT DIFFERENT FROM NORMAL KERATINOCYTES IN VITRO" was published in 2009. Journal: Indian J Dermatol.

# CELL PROLIFERATION AND CYTOKINE INDUCTION BY TNF-α OF PSORIATIC KERATINOCYTES ARE NOT DIFFERENT FROM NORMAL KERATINOCYTES *IN VITRO*

**DOI:** 10.4103/0019-5154.55631

**Published:** 2009

**Authors:** Hidetoshi Takahashi, Hitomi Tsuji, Yoshio Hashimoto, Akemi Ishida-Yamamoto, Hajime Iizuka

**Affiliations:** *From the Department of Dermatology, Asahikawa Medical College, 2-1-1-1 Midorigaokahigashi, Asahikawa 078-8510, Japan.*

**Keywords:** *Cell proliferation*, *psoriasis*, *TNF-α*

## Abstract

**Background:**

Recent studies indicate that various cytokines including tumor necrosis factor-α (TNF-α) play an essential role in the induction and maintenance of psoriatic lesion.

**Aims:**

To compare the cell proliferation of keratinocytes by various cytokines and TNF-α-induced cytokine secretion among normal keratinocytes, uninvolved, and involved keratinocytes.

**Methods:**

The keratinocytes from normal skin, uninvolved, and involved psoriasis were cultured in the presence of IL-6, IL-8, epidermal growth factor (EGF), hepatocyte growth factor (HGF), transforming growth factor-α (TGF-α) epiregulin, amphiregulin, and TNF-α and then MTT assay for keratinocytes proliferation was performed. Furthermore, TNF-α-induced secretion of IL-6, IL-8, EGF, HGF, TGF-α, epiregulin, and amphiregulin were compared among these keratinocytes.

**Results:**

IL-6, IL-8, EFG, TGF-α, epiregulin, and amphiregulin, but not TNF-α increased keratinocyte proliferation of normal, psoriatic uninvolved, and involved skin. The increased cell proliferation by these cytokines and growth factors were not different among the keratinocytes derived from normal skin, uninvolved, and involved psoriasis. The significant induction of TNF-α increased IL-6, IL-8, EGF, HGF, TGF-α, epiregulin, and amphiregulin, but the increase in these cytokines and growth factors were not different among normal skin, uninvolved, and involved psoriasis.

**Conclusion:**

Cell proliferation by various cytokines and growth factors and TNF-α-induced cytokine secretion are not different between normal and psoriatic keratinocytes.

## Introduction

Psoriasis has been characterized by hyperproliferation accompanied by acanthosis and aberrant differentiation of keratinocytes. Although the precise mechanism of hyperproliferation in psoriasis is still unclear, several growth factors and cytokines, such as epidermal growth factor (EGF), amphiregulin, epiregulin, IL-6, and IL-8, are assumed to be important.[1] Furthermore, it is supposed that TNF-α and INF-α, which are derived from dendritic cells and T cells, regulate the expression of these growth factors and cytokines. Because cyclosporine and anti-TNF-α agents, such as infliximab, adalimumab, and eternercept, are effective for psoriasis,[2] the trigger of keratinocytes hyperproliferation is presumed to be cellular immune response mediated by T cells and dendritic cells.[3] However, it is still unclear whether the keratinocytes derived from psoriasis are inherently distinct from normal keratinocytes. In the present study, we compared cell proliferation induced by various cytokines and growth factors as well as TNF-α-induced secretion of cytokine/growth factors among keratinocytes from normal skin, uninvolved, and involved psoriasis.

## Materials and Methods

### Patients

Skin samples were collected from five psoriasis (36 to 55 years old) patients and five healthy individuals (28 to 48 years old) who underwent plastic surgery. All patients had untreated, moderate to severe plaque type psoriasis. The skin was obtained after informed consent and with the approval of the Ethical Committee of the Asahikawa Medical College.

### Cell culture

Primary keratinocytes were obtained from normal, psoriatic involved, and uninvolved skin by minor modifications of the methods of Nickoloff *et al*.[4] Briefly, dermal-epidermal separation was achieved by incubation in Dulbecco's-modified Eagle's minimal essential medium supplemented with 1% dispase. The epidermis was treated with 0.25% trypsin/0.02% EDTA for 15min at 37°C. Then the keratinocytes were cultured in keratinocytes growth medium (KGM) containing insulin (5μg/ml), and bovine pituitary extract (50μg/ml) at 37°C in air containing 5% CO_2_. The calcium concentration in the medium was 0.1 mM. The keratinocytes were maintained in a subconfluent state by subculturing in every 4-5 days and various assays were performed.

### MTT assay for keratinocytes proliferation

The primary keratinocytes obtained were cultured in 96-well microtiter plates (1 × 10^3^ cells/well), and incubated for 24 h with the indicated concentrations of cytokines: TNF-α (1ng/ml), EGF (10 ng/ml), amphiregulin (1 ng/ml), hepatocyte growth factor (HGF) (10 ng/ml), epiregulin (10 ng/ml), transforming growth factor-α (TGF-α) (1 ng/ml), IL-6 (0.5 ng/ml), and IL-8 (0.5 ng/ml)). These concentrations were chosen to obtain the maximal effect on keratinocyte cell proliferation (data not shown). Non-radioactive MTT proliferation assay using tetrazolium was performed according to the protocol equipped with the assay kit, which was purchased from Promega (Madison, WI, USA).

### Cytokines assay

The primary keratinocytes obtained were cultured in 96-well microtiter plates (1 × 10^3^ cells/well), and incubated for 24 h in the presence of TNF-α (1μg/ml). Then supernatants of culture medium was collected and IL-6, IL-8, EGF, HGF, TGF-α, epiregulin, and amphiregulin were measured by enzyme-linked immunosorbent assay (ELISA) kits (BioSource). These assays detected only human cytokines and the minimal detectable concentrations were 2.4 pg/ml for TNF-α, 1.5 pg/ml for IL-6, 1.5 pg/ml for IL-8, 3.0 pg/ml for EGF, 50 pg/ml for HGF, 0.2 pg/ml for epiregulin, and 0.25 pg/ml for amphiregulin, respectively.

### Statistics

Statistical significance of the data obtained was evaluated by Student's *t*-test using unpaired analyses.

### Materials

Dulbecco's modified Eagle's medium and KGM medium were purchased from GIBCO (Grand Island, NY, USA). Penicillin and streptomycin were obtained from M.A. Bioproducts (Walkersville, MD, USA). All other chemicals were purchased from Nakarai Chemicals Ltd. (Kyoto, Japan).

## Results

### Cell growth of primary keratinocytes in the presence of various cytokines

The effect of various cytokines and growth factors on the growth of primary keratinocytes of normal (NK), psoriatic involved (PIK), and uninvolved skin (PUK) was determined. IL-6, IL-8, EGF, HGF, TGF-α, epiregulin, and amphiregulin but not TNF-α significantly increased cell proliferation of these keratinocytes [Figure 1]. The increased cell proliferation was most potent in EGF-treated keratinocytes. The increased cell proliferation by these cytokines and growth factors were not different among NK, PIK, and PUK [Figure 1].

**Figure 1:** The effect of TNF-α, IL-6, IL-8, EGF, HGF, TGF-α, epiregulin, and amphiregulin for keratinocyte cell growth (NK, PIK, and PUK (*n* = 5) were treated with TNF-α(1ng/ml), EGF (10ng/ml), amphiregulin (1ng/ml), hepatocyte growth factor (HGF) (10ng/ml), epiregulin (10ng/ml), transforming growth factor-α (TGF-α) (1ng/ml), IL-6 (0.5 ng/ml), IL-8 (0.5 ng/ml) for 24 h, and MTT assay were performed. Blue box, red box, and yellow box indicate NK, PUK, and PIK, respectively)

### Cytokines and growth factors secretion of TNF-α-treated keratinocytes

The effect of TNF-α on cytokines and growth factors secretion of keratinocytes was determined. TNF-α significantly induced the secretion of IL-6, IL-8, EGF, HGF, TGF-α, epiregulin, and amphiregulin up to 2–8-fold after 24 h [Figure 2]. The effect was observed up to 48 h (data not shown). The increased levels of cytokines and growth factors by TNF-α were not different among NK, PIK, and PUK [Figure 2].

**Figure 2:** The effect of IL-6, IL-8, EF, HGF, TGF-α, epiregulin, and amphiregulin induction in TNF-α-stimulated keratinocytes (NK, PIK, and PUK (*n* = 5) were treated with TNF-α(1 ng/ml) for 24 h, then the supernatants were collected and IL-6, IL-8, EGF, HGF, TGF-α, epiregulin, and amphiregulin assays were performed. The level of these cytokines/growth factors of untreated NK was designated as 1.0 and relative intensity was calculated. Dark blue box, red box, yellow box, and light blue indicate NK, TNF-α treated-NK, -PUK, and -PIK, respectively)

## Discussion

Psoriatic hyperproliferative epidermis has been characterized by increased keratinocyte proliferation accompanied by characteristic histopathology.[5,6] The induction of increased keratinocytes is induced by several growth factors and cytokines, such as, EGF, amphiregulin, epiregulin, IL-6, and IL-8. In addition, histochemical studies have indicated the increased local levels of various cytokines.[1–3] In the present study, we showed that EGF, amphiregulin, epiregulin, IL-6, and IL-8 increased keratinocytes proliferation confirming the previous studies.

Although T cells show an essential role in the induction and maintenance of psoriasis, it is still not clear that whether the keratinocytes derived from psoriasis show distinct behavior compared to normal keratinocytes. Oyama *et al*. showed the difference of EGF receptor expression induced by IL-6 between normal and psoriatic lesional keratinocytes.[7] They suggested different EGF receptor regulatory system regarding the pathogenesis of psoriasis. Several studies revealed the lack of effect of TNF-α on proliferation and differentiation in healthy and psoriatic keratinocytes. Also studies have reported that psoriatic keratinocytes are equally responsive to the stimulatory effects of TGF-α and IL-8, but are less susceptible to IL-6.[8,9] In the present study, increased keratinocytes proliferation induced by EGF, amphiregulin, epiregulin, IL-6, and IL-8 were not significantly different among the normal, psoriatic lesional, and nonlesional keratinocytes, thereby conforming the previous studies. Furthermore, TNF-α-induced secretion of cytokines was not different among these keratinocytes. These results suggest that the keratinocytes from psoriasis do not reveal distinct behavior regarding cell proliferation and TNF-α dependent cytokine secretion at least for the tested cytokines and that for T cells and dendritic cells but not keratinocytes are more essential for the pathogenesis of psoriasis. Finally, the recent findings suggest the essential role of Th17 cells on the pathogenesis of psoriasis.[10,11] The marked increase in IL-6 secretion by keratinocytes is quite interesting, because this cytokine is required for the Th17 cell induction.[10]
